The article "A cell-permeable tool for analysing APP intracellular domain function and manipulation of PIKfyve activity" was published in 2016. Journal: Biosci Rep.

# A cell-permeable tool for analysing APP intracellular domain function and manipulation of PIKfyve activity

**DOI:** 10.1042/BSR20160040

**Published:** 2016-04-15

**Authors:** Benjamin Guscott, Zita Balklava, Stephen T. Safrany, Thomas Wassmer

**Affiliations:** * School of Life and Health Sciences, Aston University, Aston Triangle, Birmingham B4 7ET, U.K.; † School of Pharmacy, University of Wolverhampton, Wulfruna Street, Wolverhampton WV1 1LY, U.K.

**Keywords:** Alzheimer's disease, FAB1, FIG4, neurodegeneration, phosphoinositide, VAC14, vacuolar H^+^-ATPase (V-ATPase)

## Abstract

The mechanisms for regulating PIKfyve complex activity are currently emerging. The PIKfyve complex, consisting of the phosphoinositide kinase PIKfyve (also known as FAB1), VAC14 and FIG4, is required for the production of phosphatidylinositol 3,5-bisphosphate [PI(3,5)*P*_2_]. PIKfyve function is required for homoeostasis of the endo/lysosomal system and is crucially implicated in neuronal function and integrity, as loss of function mutations in the PIKfyve complex lead to neurodegeneration in mouse models and human patients. Our recent work has shown that the intracellular domain of the amyloid precursor protein (APP), a molecule central to the aetiology of Alzheimer's disease binds to VAC14 and enhances PIKfyve function. In the present study, we utilize this recent advance to create an easy-to-use tool for increasing PIKfyve activity in cells. We fused APP intracellular domain (AICD) to the HIV TAT domain, a cell-permeable peptide allowing proteins to penetrate cells. The resultant TAT–AICD fusion protein is cell permeable and triggers an increase in PI(3,5)*P*_2_. Using the PI(3,5)*P*_2_ specific GFP-ML1Nx2 probe, we show that cell-permeable AICD alters PI(3,5)*P*_2_ dynamics. TAT–AICD also provides partial protection from pharmacological inhibition of PIKfyve. All three lines of evidence show that the AICD activates the PIKfyve complex in cells, a finding that is important for our understanding of the mechanism of neurodegeneration in Alzheimer's disease.

## Abstract (precis)

In this work we developed and validated a cell permeable tool to study the intracellular function of a central molecule in Alzheimer's disease, the amyloid precursor protein. We showed that it regulates the activity of the PIKfyve kinase complex.

## INTRODUCTION

Phosphoinositides are low abundance phospholipids that are important components of eukaryotic membranes [1,2]. Their inositol ring can be phosphorylated or dephosphorylated by a large number of phosphoinositide kinases and phosphatases respectively, allowing their interconversion [2]. Phosphoinositides are known to be distributed throughout the cell in a spatially and temporally defined manner, enabling their function as regulators of signalling hubs and membrane trafficking events and by consequence their formation and breakdown is tightly regulated. To truly understand the cycle of creation and turnover of phosphoinositides, it is necessary to understand how phosphoinositide kinases and phosphatases are regulated. Deregulation of phosphoinositide metabolism has been involved in a growing number of diseases. For example, defects in the metabolism of the endosomal phosphatidylinositol 3,5-bisphosphate [PI(3,5)*P*_2_] has been shown to result in severe neurodegeneration in both mice and humans [3–6]. PI(3,5)*P*_2_ is formed by the phosphorylation of phosphatidylinositol 3-phosphate (PI3*P*) at the 5-position of the inositol ring by the PIKfyve kinase complex that in mammals consists of the kinase PIKfyve, VAC14 which functions as a scaffold for the complex and FIG4, a 5-phosphatase that also serves as co-activator of PIKfyve [7]. Loss of function mutations in any of the genes encoding the PIKfyve complex result in reduced PI(3,5)*P*_2_ levels and neurodegeneration with the formation of large vacuoles in the brains of the affected animals in combination with extensive cell death [3–5]. This form of neurodegeneration leads to the early demise of the affected animals between birth and approximately 6 weeks. In humans, mutations in the FIG4 and VAC14 encoding genes have been shown to lead to rare cases of genetic disorders, such as Charcot–Marie–Tooth syndrome type 4J (CMT4J), amyotrophic lateral sclerosis (ALS) and Yunis–Varón syndrome, confirming that the PIKfyve complex and formation of PI(3,5)*P*_2_ are crucial for the neuronal integrity and function in humans [4,6,8].

Studying the formation and function of PI(3,5)*P*_2_ has been hampered by its low abundance in cells, posing a significant challenge for its detection. This problem has been alleviated to a certain extent by the recent establishment of GFP-ML1Nx2, a PI(3,5)*P*_2_ specific probe that allows its detection in cells [9].

PI(3,5)*P*_2_ dependent effects have been revealed using loss-of-function mutations or RNAi of PIKfyve complex members [3–5,10,11]. Importantly, with the establishment of two PIKfyve inhibitors, YM201636 and Apilimod, acute inhibition of the PIKfyve kinase has become feasible, facilitating the analysis of PI(3,5)*P*_2_ functions [12,13]. However, so far it has not been possible to acutely increase PI(3,5)*P*_2_ levels. This is particularly relevant as the endogenous level of PI(3,5)*P*_2_ at steady state is very low, so being able to boost its levels experimentally would be useful to study the functional consequences of production of PI(3,5)*P*_2_. So far this has not been possible as the mechanism by which the PIKfyve complex is regulated in mammals remained unclear. However, our recent work has shown that the amyloid precursor protein (APP), a central molecule in Alzheimer's disease, binds to the VAC14 scaffold of the complex and enhances the activity of the PIKfyve complex in cells [14], providing a specific activator of this important enzyme complex. We hypothesized that fusing the APP intracellular domain (known as AICD) to a cell-permeable peptide would allow us to generate an activator of the PIKfyve complex that can be applied exogenously to cells, and following cell penetration, would result in acute activation of PIKfyve.

The creation of cell-penetrating peptides has been enabled by the discovery that the HIV TAT protein is transduced into cells by a mechanism that still remains ill characterized [15,16]. Based on this discovery, a number of cell-penetrating peptides have been established [17]. In the present study, we utilized the HIV TAT domain (YGRKKRRQRRR) to allow AICD to penetrate cells and test whether this would alter PIKfyve activity. We show that AICD fused to the TAT domain is indeed able to successfully penetrate cells and that TAT–AICD leads to an increase in PI(3,5)*P*_2_. We confirm the increased PIKfyve activity using the PI(3,5)*P*_2_ probe ML1Nx2. TAT–AICD also confers partial resistance to pharmacological PIKfyve inhibition. All three lines of evidence establish TAT–AICD as an easy-to-use tool for exogenous activation of PIKfyve and more generally for studying the function of the AICD.

In light of the recent controversy concerning the suggested regulation of the vacuolar H^+^-ATPase (V-ATPase) by PI(3,5)*P*_2_ [18,19], we also analysed whether PIKfyve inhibition has an impact on the endo/lysosomal acidification. We found that both PIKfyve inhibitors, YM201636 and Apilimod, significantly reduced the number of lysotracker and LampI positive vesicles, suggesting that PIKfyve does regulate important aspects of endo/lysosomal acidification through a yet unclear mechanism.

## MATERIALS AND METHODS

### Antibodies, lysotracker and PIKfyve inhibitors

Mouse monoclonal anti-LampI (clone H4A3) antibody (sc-2001) was obtained from Santa Cruz Biotechnology. Mouse monoclonal anti-maltose-binding protein (MBP) antibody (E8032) and anti-mouse Alexa 555 secondary antibody (4409S) were purchased from New England Biolabs. Lysotracker DND-99 (L-7528) was purchased from Thermo Fisher. YM201636 was purchased from Abcam (ab141370), Apilimod from US Biological (002800).

### DNA manipulations and construction of His–MBP–TAT–AICD and His–MBP–TAT

The expression plasmid for His–MBP–TAT–AICD was based on pET28-MBP-TEV established in [20]. The 47 amino acid encoding DNA fragment of AICD was PCR amplified with a TAT domain encoded in the 5'-primer of the PCR product. This primer introduced the TAT sequence between MBP and AICD as indicated in the scheme in Figure 1(A), with a HindIII site separating TAT from AICD. This fragment was cloned with BamHI (5') and XhoI (3') into pET28-MBP-TEV to result in an in frame fusion with MBP, termed pET28-MBP–TAT–AICD. Plasmid pET28-MBP-TAT for expression of the His–MBP–TAT control protein was created by HindIII digest of pET28-MBP–TAT–AICD and filling in of the cohesive ends of the HindIII site using the Pfu polymerase and religation, thus introducing four additional bases, resulting in a frame shift eliminating AICD expression. The expression construct for pET28-MBP–AICD was described in [21].

**Figure 1:** Construct design and purification of His–MBP–TAT, His–MBP–TAT–AICD and His–MBP–AICD (**A**) Schematic representation of the fusion proteins designed in the present study. The 6xHis tag was introduced for Ni-affinity chromatography. The MBP strongly enhances the solubility of the purified proteins. The cell-penetrating TAT motif was introduced at the C-terminus of MBP to allow the transport of the protein inside the cell. Two negative controls were utilized: One lacking the AICD domain, controlling for AICD independent effects, one lacking the TAT domain, precluding its entry into the cell and controlling for potential extracellular effects. (**B**) Coomassie stained gel of 1 μg of the purified proteins. Although a minor degradation product of the His–MBP–TAT–AICD protein is visible, most of the preparation represents the full length protein, indicated by the slightly higher apparent molecular mass compared with the control proteins His–MBP–TAT and His–MBP–TAT–AICD.

### Protein expression and purification

His–MBP–TAT, His–MBP–TAT–AICD and His–MBP–AICD were expressed as described in [21]. Purified proteins (concentrations ranged from 2.5 to 3.5 mg/ml) were dialysed against 25 mM Hepes, pH 7.2, 125 mM potassium acetate, 1 mM EDTA.

### Cell culture transfections

HeLa cells were grown in DMEM containing 10% foetal calf serum and 1x penicillin/streptomycin. HeLa cells were seeded on to glass coverslips in a 24-well plate at a density of 100000 cells per well and incubated at 37°C with 5% CO_2_ overnight. The following day, the cells were transfected with the pEGFP-c3-ML1Nx2 plasmid using Lipofectamine 2000 according to the manufacturer's protocol. Cells were utilized for experiments the following day.

### Immunostaining and fluorescence microscopy

HeLa cells were fixed for 20 min in 4% formaldehyde (from depolymerized paraformaldehyde) in PBS, followed by two washes in PBS. Cells were permeabilized using 0.1% Triton X-100 in PBS for 4 min followed by two washes in PBS and blocking using 2% BSA in PBS for at least 15 min. Cells were stained by use of a primary antibody (diluted 1/300 for anti-LampI and 1/200 for anti-MBP in PBS containing 2% BSA, incubation for 1 h at room temperature) followed by three washes in PBS and incubation with the secondary antibody (diluted 1:500 in 2% BSA in PBS, incubation for 1 h, room temperature). Finally, cells were washed thrice using PBS and mounted using Mowiol. Samples were imaged on a Leica SP5 TCS II MP confocal microscope with a 63× oil immersion lens.

### Protein uptake assay

HeLa cells, were seeded the previous day at 100000 cells/ml in 24-well plates on coverslips. Cells were treated with 350 nM or 700 nM of either MBP-AICD, MBP-TAT or MBP-TAT–AICD diluted in standard growth medium (DMEM with 10% foetal calf serum and 1x penicillin/streptomycin) and added to cells, followed by incubation for 60 min in a tissue culture incubator. Cells were either fixed for 20 min using 4% formaldehyde and mounted using Mowiol or immunostained.

### Vacuole quantification

Cells were pretreated with His–MBP–TAT, His–MBP–AICD or His–MBP–TAT–AICD for 1 h, followed by addition of 1 μM YM201636 for 45 min before fixation in 4% formaldehyde in PBS. Fixed cells were imaged using a Nikon Eclipse TS100 inverted microscope under a 40× objective. Vacuolar structures in each cell of a sample (first five cells per image, top left to right) were counted and used to quantify the structures per cell for each condition. One-way ANOVA (*α*=0.05) was performed in GraphPad Prism 6.

### Biochemical quantification of phosphoinositides

Cells (2×10^5^/well of a six-well plate) were labelled with 50 μCi/ml *myo*-[^3^H]inositol (ARC) in 2 ml inositol-free DMEM (MPBio), supplemented with L-glutamine and dialysed foetal calf serum (10%, Gibco Life Technologies) for 96 h, prior to addition of His–MBP–TAT, His–MBP–AICD or His–MBP–TAT–AICD (700 nM) for 1 h. The reaction was quenched by the removal of the medium and addition of 0.6 M HClO_4_. Inositol lipids were extracted from the HClO_4_ pellet and prepared as previously described [22] and analysed using a modified gradient: samples in water were loaded on to a Partisphere (5 μm) SAX column equipped with matching guard cartridge (HiChrom) eluted with the following gradient to 1.0 M (NH_4_)H_2_PO_4_, adjusted to pH 3.8 with H_3_PO_4_ (B), at a flow rate of 1.0 ml/min: 0 min, 0% B; 5 min, 0% B; 91 min, 30% B; 126 min, 100% B. Fractions (1 ml) were collected, mixed with 2.5 ml Proflow P+ scintillant (Meridian) and assessed for radioactivity. Peaks were ascribed by co-elution of standards in parallel runs.

### Lysotracker staining

HeLa cells were seeded at a density of 100000/ml in 24-well plates on coverslips. The following day cells were treated with either 0 nM, 25 nM or 250 nM Apilimod, 100 nM or 1 μM YM201636 or 10 mM ammonium sulfate for 4 h. One micromolar lysotracker Red was added to cells for 5 min, followed by fixation with 4% formaldehyde in PBS, washed twice with PBS and mounted using Mowiol.

### Automated quantification of vesicles for analysing GFP-ML1Nx2, lyostracker and LampI

Using the Fiji version of ImageJ maximum *z*-projections were created with a black mask excluding non-quantified cells, an image of which was exported for future reference. Each cell underwent automated Squassh analysis using the MOSAIC suite in ImageJ as described recently [14,23]. Object data collected from the analysis were exported to LibreOffice Calc where a threshold for structure size was implemented–only structures over 1 pixel in size and over 0.15 average intensity were included in the analysis to exclude background noise introduced by the confocal detector. Statistical analysis was performed using one-way ANOVA with Tukey's post-hoc test in GraphPad Prism 6 (*α*=0.05).

## RESULTS

First we tested whether fusion of the TAT domain to the AICD would enable effective protein transduction into the cytoplasm of tissue culture cells. We fused the HIV TAT domain, the first well established cell-penetrating peptide [15,16], to the N-terminus of AICD. As a control protein we created His–MBP–TAT, identical in design to His–MBP–TAT–AICD but lacking AICD. This fusion protein should allow us to control for any effects the other domains (e.g. 6xHis tag, MBP, TAT) may have inside the cell. As a second negative control, we utilized the recently established His–MBP–AICD [21] that, lacking a cell-penetrating motif, should be unable to enter cells (Figure 1A). All three proteins were expressed in *Escherichia coli*, purified by nickel affinity chromatography and analysed for purity and integrity (Figure 1B). All three proteins were successfully purified (total yield ≥10 mg from 0.5 L expression culture). A minor degradation product was detected for His–MBP–TAT–AICD, presumably by proteolytic cleavage at the C-terminus of the construct, as we utilized an N-terminal His tag for purification. However, the vast majority of the purified protein in the sample appeared to be full length and thus was deemed suitable for use in our assays.

We tested whether the purified proteins were able to penetrate HeLa cells using either 350 nM or 700 nM. The fusion proteins were added to normal growth medium for 5 min, 15 min, 30 min and 60 min followed by fixation, immunostaining using an anti-MBP antibody and mounting for microscopy. Confocal imaging revealed strong labelling of cells treated with His–MBP–TAT and His–MBP–TAT–AICD, whereas no staining was visible in the His–MBP–AICD control lacking a TAT motif (Figure 2A). Three hundred and fifty nanomolars led to a very similar staining pattern as 700 nM, only slightly weaker (results not shown). These data showed that the TAT motif is necessary for MBP detection in cells, suggesting that the TAT motif indeed allowed successful cell penetration.

**Figure 2:** His–MBP–TAT and His–MBP–TAT–AICD successfully penetrate HeLa cells (**A**) A time course of protein uptake into HeLa cells for 5–60 min in which 700 nM His–MBP–TAT, His–MBP–TAT–AICD and His–MBP–AICD were added to the cells and incubated for the times indicated, followed by fixation, permeabilization and immunostaining with an anti-MBP antibody and an anti-mouse Alexa 555 secondary antibody. In His–MBP–TAT and His–MBP–TAT–AICD treated cells strong staining is visible, suggesting that the TAT domain enabled protein uptake into the cells where it was retained. The His–MBP–AICD control protein, lacking the TAT domain failed to show any appreciable staining, demonstrating that the TAT domain is necessary for cell penetration. His–MBP–TAT showed diffuse localization throughout the time course whereas His–MBP–TAT–AICD strongly localized to vesicular structures, particularly so after 30 min and 60 min. The outline of example cells is shown in white to facilitate the interpretation of the images. (**B**) HeLa cells transfected with the PI(3,5)*P*_2_ specific GFP-ML1Nx2 probe were incubated with 700 nM of the fusion proteins indicated for 30 min, followed by fixation, permeabilization and immunostaining with an anti-MBP antibody. His–MBP–TAT–AICD was found to display co-localization with the GFP-ML1Nx2 probe. (A and B) White boxes indicate the area enlarged in the inset. Scale bars, 20 μm.

Interestingly, although after 5 min of incubation the staining patterns for His–MBP–TAT and His–MBP–TAT–AICD looked similar, the patterns diverged over time. Particularly, after 30 min and 60 min, the His–MBP–TAT staining remained diffuse with the outline of cells still visible. In contrast, His–MBP–TAT–AICD showed a vesicular staining pattern, suggesting that His–MBP–TAT–AICD had reached a vesicular destination as we would expect according to our previous work (Figure 2A) [14].

Our recent work has shown that AICD binds the PIKfyve complex and stimulates the formation of PI(3,5)*P*_2_ positive vesicles [14]. Therefore we tested, whether His–MBP–TAT–AICD displayed any co-localization with the PI(3,5)*P*_2_ specific GFP-ML1Nx2 probe [9]. HeLa cells were transfected with the GFP-ML1Nx2 probe and treated for 30 min with 700 nM of the fusion proteins, followed by immunostaining with an anti-MBP antibody. Confocal microscopy showed that the His–MBP–TAT–AICD protein displayed instances of co-localization with GFP-ML1Nx2, whereas we could not detect any for the His–MBP–TAT control protein (Figure 2B). Again, no label was detected with the His–MBP–AICD control consistent with the lack of cell penetration of this protein into cells. These data suggest that at His–MBP–TAT–AICD can reach a PI(3,5)*P*_2_ positive target organelle.

Next, we tested whether His–MBP–TAT–AICD is able to modify PIKfyve activity. We measured the various phosphoinositide species biochemically by radiolabelling HeLa cells with tritiated inositol, challenging them with the three fusion proteins and analysing the impact on the various phosphoinositides using HPLC and scintillation counting [22]. We were able to detect PI3*P*, phosphatidylinositol 4-phosphate (PI4*P*), phosphatidylinositol 4,5-bisphosphate [PI(4,5)*P*_2_], phosphatidylinositol 3,4-bisphosphate [PI(3,4)*P*_2_], PI(3,5)*P*_2_ and phosphatidylinositol 3,4,5-trisphosphate [PI(3,4,5)*P*_3_]. The only species we were unable to quantify was phosphatidylinositol 5-phosphate (PI5*P*) as this could not be separated from the much more abundant PI4*P* by HPLC and is by consequence included in the PI4*P* counts. The outcome of this analysis is presented in Table 1. Phosphoinositides were normalized to the highly abundant plasma membrane phosphoinositide PI(4,5)*P*_2_. Two phosphoinositides were significantly increased in the His–MBP–TAT–AICD sample: PI(3,5)*P*_2_ and PI(3,4)*P*_2_. The significant increase in PI(3,5)*P*_2_ is entirely consistent with the idea that AICD binds the PIKfyve complex and increases its activity. What mechanism drives the increase in PI(3,4)*P*_2_ is currently unclear.

**Table 1:** Quantification of phosphoinositides in HeLa cells upon treatment with His–MBP–TAT, His–MBP–TAT–AICD and His–MBP–TAT–AICD Data are normalized to PI(4,5)*P*_2_ being 100% in each individual experiment and expressed as percentage of PI(4,5)*P*_2_ ± S.E.M, *n*=4–7. Significant differences are indicated by *P<0.05, using one-way ANOVA and Dunnett's post-hoc test performed in GraphPad Prism 6.0. PI(3,5)*P*_2_ levels are significantly increased in His–MBP–TAT–AICD treated cells compared with those treated with control proteins His–MBP–TAT and His–MBP–AICD or untreated control cells. Note that we were not able to quantify the lower abundant PI5*P* as it could not be resolved from the PI4*P* peak and is by consequence included in PI4*P*.

	Control	His–MBP–TAT	His–MBP–AICD	His–MBP–TAT–AICD
gPI3*P*	10±1.2	8.8±0.9	9±2	12±2
gPI4*P*	230±40	250±70	190±100	130±20
gPI(3,5)*P*_2_	1.4±0.4	1.3±0.4	2.2±0.2	3.3±0.4*
gPI(3,4)*P*_2_	7±3	8±4	10±4	22±3*
gPI(3,4,5)*P*_3_	5±2	4±1	7±2	10±1

Next, we tested whether His–MBP–TAT–AICD has an impact on PI(3,5)*P*_2_ using GFP-ML1Nx2. HeLa cells transfected with GFP-ML1Nx2 were challenged with 700 nM of the fusion proteins for 1 h, followed by fixation, mounting and analysis by confocal microscopy. The GFP-ML1Nx2 staining pattern was analysed using the image segmentation tool implemented in the MOSAIC suite in ImageJ. This software allows the automatic detection and characterization of vesicles in cells with minimal manual input, enabling objective analysis of the phenotype and precluding potential bias introduced by the observer [23].

Our recent work has shown that overexpression of APP and AICD both led to an increase in the number of GFP-ML1Nx2 positive vesicles [14]. Therefore, we first analysed the average number of GFP-ML1Nx2 positive vesicles per cell. Using His–MBP–TAT–AICD, we detected a significant increase in the average number of GFP-ML1Nx2 positive vesicles (Figures 3A and 3B). Compared with overexpression of APP or AICD the effect of His–MBP–TAT–AICD appeared to be relatively small, suggesting that DNA transfection of individual cells may be more effective at delivering an exogenous protein compared with utilizing a cell-penetrating peptide.

**Figure 3:** His–MBP–TAT–AICD modulates PI(3,5)*P*_2_ dynamics (**A**) HeLa cells expressing the PI(3,5)*P*_2_ probe GFP-ML1Nx2 were treated with 700 nM His–MBP–TAT, His–MBP–TAT–AICD and His–MBP–AICD for 1 h followed by fixation, mounting and confocal microscopy. Compared with the negative controls (His–MBP–TAT and His–MBP–AICD), His–MBP–TAT–AICD increased the number and size of GFP-ML1Nx2 positive vesicles. Enlargements (white boxes) are presented below the respective image. Scale bar, 20 μm. (**B** and **C**) Effect of the three proteins on GFP-ML1Nx2 (presented in A) were quantified using the MOSAIC suite in ImageJ for automatic detection of GFP-ML1Nx2 positive vesicles. Plotted are the average number of GFP-ML1Nx2 positive vesicles per cell (B) and their average size (C). Data were pooled from three independent experiments, a total of 83 cells were analysed for His–MBP–TAT, 68 cells for His–MBP–TAT–AICD and 81 cells for His–MBP–AICD. Error bars are S.E.M. (**D**) Inhibition of PIKfyve using YM201636 for 45 min led to the formation of vacuoles detectable by light microscopy. It was tested whether His–MBP–TAT, His–MBP–TAT–AICD or His–MBP–AICD could modify the sensitivity of HeLa cells to PIKfyve inhibition. His–MBP–TAT–AICD reduced the appearance of vacuoles compared with the two control proteins. Arrows indicate examples of vacuoles. Scale bar, 100 μm. (**E**) Quantification of the average number of vacuoles per cell upon PIKfyve inhibition. His–MBP–TAT–AICD significantly reduced the average number of vacuoles per cell compared with the negative controls, His–MBP–TAT and His–MBP–AICD. Note that vacuoles are not detectable in the absence of PIKfyve inhibition. A total of 150 cells per condition were analysed collected in three independent experiments. Error bars are S.E.M. Statistical analysis in (B), (C) and (E) was performed using one-way ANOVA with Tukey's post-hoc test, *α*=0.05, **P≤0.01, ****P≤0.0001.

We also noted that the average size of GFP-ML1Nx2 positive vesicles was increased compared with the two negative controls (Figure 3C). Thus, His–MBP–TAT–AICD is able to increase both the number and size of PI(3,5)*P*_2_ positive vesicles, entirely consistent with the idea that the AICD can modulate PIKfyve activity.

Inhibition of PIKfyve using various means is well known to result in the formation of vacuoles, aberrant structures that are derived from the endosomal system [3,11,24]. If AICD is able to stimulate PIKfyve activity then it may be able to mitigate the effect of pharmacological PIKfyve inhibition. We tested this idea by pretreating HeLa cells with the three fusion proteins, followed by PIKfyve inhibition using 1 μM YM201636 for 45 min. After fixation, the number of vacuoles in cells was counted. Treatment of cells with His–MBP–TAT–AICD significantly reduced the average number of vacuoles per cell compared with the negative controls His–MBP–TAT and His–MBP–AICD (Figures 3D and 3E), suggesting that application of His–MBP–TAT–AICD indeed provided partial protection from PIKfyve inhibition.

Taken together these findings show that His–MBP–TAT–AICD is able to activate the PIKfyve complex, confirming and extending our previous work. These data establish His–MBP–TAT–AICD as a user friendly tool to acutely activate the PIKfyve complex.

### Dependence of acidification of endo- and lysosomes on PIKfyve

Recent work from the Kane lab suggested that FAB1, the yeast orthologue of PIKfyve, is able to regulate the assembly state of the V-ATPase [18] in yeast, a proton pump that controls acidification of yeast vacuoles, organelles equivalent to lysosomes in metazoa. However, Ho et al. [19] found that under steady state conditions mutation of *fab1* did not seem to affect vacuolar pH. Interestingly though, FAB1 played a role in adaptation of the vacuolar pH in response to osmotic shock, known to strongly stimulate PIKfyve activity [25]. These observations would suggest that FAB1/PIKfyve can, at least under certain conditions, affect vacuolar acidification although it may be dispensable for controlling the luminal pH of vacuoles under steady state conditions. The situation in mammalian cells is currently not clear. Ho et al. found in RAW macrophages in which PIKfyve was inhibited using either 20 nM Apilimod or 1 μM MF4 (structurally similar to YM201636) that lysotracker staining could still be detected in vacuolar structures; however, it was restricted to the rim of vacuoles. Additionally, Ho et al. [19] found that endo/lysosomal pH appeared to be unaffected by PIKfyve inhibition using ratiometric pH detection with FITC dextran.

As the question whether PIKfyve controls endo/lysosomal acidification is important, we attempted to clarify whether this depends on PIKfyve. We utilized lysotracker DND-99 to analyse acidification of organelles and performed PIKfyve inhibition using Apilimod at 25 nM and 250 nM for 4 h. From the lysotracker staining it was evident that small, acidic vesicles remained in the cytoplasm of PIKfyve inhibited cells, consistent with the analysis of Ho et al. [19]. However, there was a marked reduction in their number. Using image segmentation, we automatically detected and quantified the average number of lysotracker positive vesicles in cells and found them to be reduced by approximately 50% with both Apilimod concentrations (Figures 4A and 4B). We also noted a slight decrease in the average vesicle intensity using 25 nM Apilimod and a somewhat more pronounced reduction using 250 nM Apilimod (Figure 4C). It should be noted that under both conditions there is abundant vacuole formation apparent under the light microscope, particularly using the higher Apilimod concentration (results not shown). However, we did not detect significant lysotracker staining in these vacuoles. This seems to be an important difference between the RAW macrophage line and HeLa cells utilized in the present study.

**Figure 4:** Inhibition of PIKfyve using Apilimod affects the number of acidified organelles and LampI positive late endosomes and lysosomes (**A**) Inhibition of PIKfyve using two different concentrations of Apilimod (25 nM and 250 nM) led to a strong decrease in the number of acidified organelles labelled with lysotracker Red DND-99. (**B**) Quantification of the average cellular number of lysotracker positive vesicles measured using Squassh analysis in the MOSAIC suite in ImageJ. Both 25 nM and 250 nM Apilimod significantly reduced the number of lysotracker positive vesicles. (**C**) Quantification of average vesicular lysotracker intensity showed a small but significant reduction in vesicular lysotracker staining with 25 nM Apilimod and a stronger reduction with 250 nM. (A–C) Data were pooled from three independent experiments, yielding a total of ≥309 cells per condition. Error bars are S.E.M. (**D**) Analysis of the LampI positive compartment upon inhibition of the PIKfyve complex using 25 nM and 250 nM Apilimod. Both concentrations of Apilimod reduced the number of LampI positive vesicles. (**E**) Quantification of the average number of LampI positive vesicles per cell and its dependence on PIKfyve showed that its inhibition reduced the number of LampI positive late endosomes and lysosomes. (**F**) Analysis of average size of LampI positive late endosomes/lysosomes showed that although the number of LampI vesicles per cell was reduced, their size increased, suggesting swelling or aggregation of the compartment. Data presented in (E) and (F) were pooled from three independent experiments with 240 cells analysed per condition. Error bars are S.E.M. Statistical analysis in (B), (C), (E) and (F) was performed using one-way ANOVA with Tukey's post-hoc test, *α*=0.05, ***P≤0.001, ****P≤0.0001.

The reduction in the number of lysotracker positive vesicles upon PIKfyve inhibition could be explained either by (A) reduced acidification of endo/lysosomes or (B) a reduction in the number of late endosomes or lysosomes. To investigate this more closely, we analysed the LampI-positive compartment and how it reacts to PIKfyve inhibition using 25 nM or 250 nM Apilimod for 4 h. Interestingly, the number of LampI positive vesicles was also reduced by approximately 50%, mirroring the effect seen with lysotracker staining. We additionally noticed an increase in the average size of LampI positive vesicles, suggesting that the compartment may either swell or aggregate, possibilities we could not differentiate by light microscopy. It should be noted that in HeLa cells, in our hands the rim of large vacuoles is almost never LampI positive. In contrast, we detect small LampI positive vesicles in close proximity to enlarged vacuoles, whereas Li et al*.* [9] showed very clear mCherry–LampI localization to the membrane of these. Currently, it is unclear whether the difference stems from the different cell models used (HeLa compared with COS1) or whether from endogenous compared with overexpressed LampI.

To test whether the observed effect on acidification as analysed by lysotracker staining is indeed PIKfyve specific, we also utilized YM201636 at 100 nM and 1 μM for 4 h. YM201636 also reduced the number of lysotracker positive vesicles. The effect was less pronounced than with Apilimod (Figures 5A and 5B), entirely consistent with our experience with the two PIKfyve inhibitors in which Apilimod consistently leads to a stronger phenotype than YM201636. We also used ammonia, a weak base that is trapped in acidic compartments and thereby reduces the concentration of free protons, increasing the organellar pH [26]. As expected the addition of 10 mM ammonium sulfate for 4 h strongly decreased the number of acidified vesicles in cells (Figures 5A and 5B), confirming that lysotracker truly labelled acidified compartments.

**Figure 5:** Effect of PIKfyve inhibition with YM201636 on acidic compartments (**A**) Lysotracker staining revealed that PIKfyve inhibition using YM201636, similar to Apilimod, reduced the average number of acidified vesicles in cells. The effect observed was weaker than with Apilimod which is consistent with the lower potency of YM201636. Inhibition of acidification using the weak base, ammonia also reduced the number of lysotracker positive vesicles, confirming that the lysotracker probe utilized indeed reflected acidification. (**B**) Quantification of the number of lysotracker positive vesicles. Data were pooled from three independent experiments, a total of 240 cells per condition were analysed for control and YM201636 samples, whereas 104 cells were analysed for ammonium sulfate treatment. Error bars are S.E.M. Statistical analysis was performed using one-way ANOVA with Tukey's post-hoc test, *α*=0.05, ***P≤0.001, ****P≤0.0001.

Taken together these data suggest that inhibition of PIKfyve affects the formation or maintenance of acidic compartments in HeLa cells.

## DISCUSSION

In the present study, we established His–MBP–TAT–AICD as a convenient, cell-permeable tool for studying the function of the AICD. Using this novel tool, we showed that His–MBP–TAT–AICD is able to activate the PIKfyve complex in cells (1) by measuring PI(3,5)*P*_2_ levels biochemically, (2) using a fluorescent PI(3,5)*P*_2_ specific probe and (3) in a functional assay where His–MBP–TAT–AICD partially suppressed the vacuole phenotype of pharmacological PIKfyve inhibition. These data are in full agreement with our recent work that showed that APP binds VAC14 of the PIKfyve complex and that this binding translates into increased PIKfyve activity [14]. This interplay is likely to be conserved throughout the metazoan evolution, as we have shown that the APP orthologue genetically interacts with the PIKfyve complex in *Caenorhabditis elegans* [21].

In the present study, we provide a much needed tool for studying APP-dependent signalling transduction mechanisms. APP has previously been suggested to engage in cell signalling. It was suggested to regulate gene expression in a fashion similar to Notch, where cleavage by β- and γ-secretase liberates the Notch intracellular domain, allowing it to translocate to the nucleus and control transcription [27], a mechanism still controversially discussed in the case of APP. Using His–MBP–TAT–AICD will facilitate the study of APP's role in transcription regulation and allow us to study functions driven by AICD.

The system presented here has two significant advantages over previous, transfection-based delivery of AICD. First, we observed virtually complete penetrance of the HeLa populations studied by our TAT containing fusion proteins. Throughout our experiments, we failed to detect cells that had not taken up the TAT fusion protein. This represents a clear advantage over plasmid based overexpression where cell penetrance can range, depending on the quality transfection reagent, from very low to acceptable. This advantage will improve biochemical studies of AICD function where low penetrance may lead to ambiguous results. Second, this system allows acute introduction of AICD which is not possible with transfection based protein expression where usually at least 24 h pass between transfection and analysis of the phenotype, during which transcription and translation gradually increase the protein level.

One current limitation of the His–MBP–TAT–AICD fusion protein is its suboptimal performance in immunofluorescence microscopy. In our hands, TAT-motif containing proteins strongly adhere not only to cells but also to the glass surface of the cover slip, resulting in strong background fluorescence in widefield microscopy. This problem can be mitigated somewhat using confocal microscopy, however, ultimately the goal will be to eliminate this binding by using a different support surface for cells other than glass or, alternatively, by coating the coverslips.

A second, more significant caveat of using the His–MBP–TAT–AICD fusion in the study of PIKfyve function is the unexpected rise of PI(3,4)*P*_2_ levels. A large body of work has shown that PIKfyve is undoubtedly a 5-kinase, by consequence there is no reason to suspect that PIKfyve is implicated in the increase in PI(3,4)*P*_2_, generated by the activity of phosphatidylinositide 4-kinases (PI4Ks). Whether APP can activate PI4Ks directly or indirectly via its intracellular domain will need to be explored in future work. It will be interesting to see whether this activity can be narrowed down to a specific motif in AICD and thus potentially separated from the effect on PI(3,5)*P*_2_ via PIKfyve.

Development of exogenous activators of the PIKfyve complex is important not only as a research tool but for the treatment of human diseases. It is extremely well documented that dysfunction of the PIKfyve complex can lead to serious neurodegenerative diseases, including CMT4J, ALS and the more recently described Yunis–Varón syndrome [3,6,8]. Loss of function mutations in a downstream effector of PIKfyve, the TRP channel TRPML-1 (also known as mucolipin-1) leads to mucolipidosis type IV, entailing developmental delays, psychomotor abnormalities, intellectual disability and a shortened lifespan [28]. Taken together these genetic diseases highlight the significance of the PIKfyve pathway for neuronal function and integrity.

Our work has shown that the central molecule in Alzheimer's disease, APP, binds to and activates the PIKfyve complex [14]. A significant body of literature has established that APP is aberrantly processed in Alzheimer's disease. This led us to propose that aberrant cleavage of APP is likely to affect PIKfyve activity which could result in neurodegeneration in Alzheimer's disease driven by reduced levels of PI(3,5)*P*_2_ [14,21,29]. If this model is correct then exogenous activation of the PIKfyve complex should mitigate or stop neurodegeneration in Alzheimer's disease. Thus, an exogenous activator of the PIKfyve complex, expected to be beneficial in PIKfyve associated genetic diseases, may also be effective in Alzheimer's disease. The development of His–MBP–TAT–AICD demonstrates that exogenous activation of PIKfyve is feasible at least in principle. It raises the possibility that a similar function could be achieved using a small molecule activator for PIKfyve that is more clinically suited.

Although the number of PIKfyve effectors is slowly growing, there is still a dearth of information on the pathways that are regulated by PI(3,5)*P*_2_. Elucidation of these pathways is necessary for us to better understand how PIKfyve dysfunction induces neurodegeneration and other defects in peripheral tissues such as bone. In this light the study suggesting that the V-ATPase is regulated by FAB1/PIKfyve is interesting [18], as the V-ATPase is important for the function of the endo/lysosomal system. Whereas data from the Kane lab suggested that FAB1 controls the assembly state of the V-ATPase in yeast, the Botelho lab found that in *fab1* mutants the vacuolar pH is unaltered at steady state. However, the pH of *fab1* mutant cells increased more rapidly in response to a hyperosmotic shock than in wild-type controls [19]. This would suggest that FAB1/PIKfyve controls the vacuolar pH at least when exposed to a hyperosmotic shock which is well known to lead to a rapid burst of PI(3,5)*P*_2_ production [25]. When studying the macrophage RAW cell line, Ho et al*.* [19] did not find any significant effect of PIKfyve inhibition on endo/lysosomal pH analysing individual endo/lysosomes.

Using the HeLa model we found that PIKfyve inhibition, using two different inhibitors at different concentrations, resulted in a reduction in the number of acidic structures per cell. This would suggest that PIKfyve plays a role in maintaining acidified organelles. It is important to note that the data of Ho et al. [19] are not directly comparable with our data in which we analysed the number of acidified organelles per cell rather than the acidification state of individual organelles.

Although our data suggest that PIKfyve has an impact on the number of acidified organelles, we currently cannot say by which mechanism. It could be a direct effect as suggested by the Kane lab in which PI(3,5)*P*_2_ produced by PIKfyve controls the assembly state of the V-ATPase and by consequence controls the pH of endo/lysosomes. Another option is that PIKfyve controls the flow of membranes to the late endosome and lysosome. This flow may regulate the number of endo- and lysosomes in the cell. PIKfyve was suggested to control maturation from early to late endosomes and to control the fission and fusion cycle of these via TRPML-1 [30–32]. The fact that PIKfyve inhibition reduced the number of LampI positive endo- and lysosomes would be consistent with this idea. Regardless of the mechanism, PIKfyve seems to have an impact on the number of acidified organelles in the cell and therefore on the cellular capacity to down-regulate certain biomolecules in lysosomes [14].

It will be important to analyse the impact of PIKfyve inhibition on the endosomal system in greater detail in future work if we are to establish which aspects of endo/lysosomal dysfunction lead to the profound neurodegeneration observed in patients with PIKfyve pathway deficiency.

## Abbreviations

AICD: APP intracellular domain
ALS: amyotrophic lateral sclerosis
APP: amyloid precursor protein
CMT4J: Charcot–Marie–Tooth syndrome type 4J
MBP: maltose-binding protein
PI4K: phosphatidylinositide 4-kinase
PI3*P*: phosphatidylinositol 3-phosphate
PI4*P*: phosphatidylinositol 4-phosphate
PI5*P*: phosphatidylinositol 5-phosphate
PI(3: 4)*P*_2_, phosphatidylinositol 3,4-bisphosphate
PI(3: 5)*P*_2_, phosphatidylinositol 3,5-bisphosphate
PI(4: 5)*P*_2_, phosphatidylinositol 4,5-bisphosphate
V-ATPase: vacuolar H^+^-ATPase
